# Long non-coding RNA FEZF1-AS1 promotes the proliferation and metastasis of hepatocellular carcinoma via targeting miR-107/Wnt/β-catenin axis

**DOI:** 10.18632/aging.202960

**Published:** 2021-05-23

**Authors:** Jing Yao, Zhe Yang, Jun Yang, Zhi-Gang Wang, Zheng-Yun Zhang

**Affiliations:** 1 Department of Surgery, Shanghai Jiao Tong University Affiliated Sixth People’s Hospital, Shanghai 200233, China

**Keywords:** hepatocellular carcinoma, lncRNA FEZF1-AS1, miR-107, β-catenin

## Abstract

Hepatocellular carcinoma (HCC) is a public health problem around the world, with the molecular mechanisms being still incompletely clear. This study was carried out to explore the role and mechanism of long-noncoding RNA (lncRNA) FEZF1-AS1 in HCC progression. RNA sequencing and quantitative real time polymerase chain reaction (qRT- PCR) were applied to identify differently expressed lncRNAs in HCC tissues and adjacent normal tissues. CCK8 assay was adopted to test cell proliferation and flow cytometry was taken to detect cell apoptosis. Wound healing assay and transwell experiment were performed to determine cell migration and invasion. To validate the function of lncRNA FEZF1-AS1 *in vivo*, tumor-burdened models were established. The results showed that lncRNA FEZF1-AS1 level was prominently enhanced in HCC tumor specimens and overexpression of FEZF1-AS1 promoted the proliferation, migration and invasion of HCC cells. In mechanism, overexpression of FEZF1-AS1 reduced the expression of miR-107 which inhibited the activation of Wnt/β-catenin signaling. Overexpression of β-catenin promoted cell proliferation, migration and invasion which were inhibited by FEZF1-AS1 downregulation. In conclusion, our study demonstrated that FEZF1-AS1 promoted HCC progression through activating Wnt/β-catenin signaling by targeting miR-107, which provided a novel target for the therapy of HCC.

## INTRODUCTION

Hepatocellular carcinoma (HCC) is a leading cause of cancer death. It is the main type of primary liver cancer [1, 2]. Although HCC therapy is in fast development, such as tissue resection, liver translation, chemotherapy, radiotherapy and biotherapy, patients with HCC still present with unfavorable prognosis and low 5-year survival rates [3, 4]. In recent years, the molecular mechanisms underlying HCC have attracted more and more attentions, and many genes play a critical role in HCC development [5]. However, it’s still a long road to elucidate fully the molecular mechanisms of HCC. It is of significance to find novel biological markers for the diagnosis and treatment of HCC.

Lots of long-noncoding RNAs (lncRNAs) were found to be oncogenes and tumor suppressors in many tumors by regulating the translation of RNA and transcription of DNA [6, 7]. For example, lncRNA GNAT1-1 was identified as a tumor suppressor in colorectal cancer by regulating the RKIP/NF-kB/Snail signaling [8]. In addition, LL22NC03-N64E9.1 was identified as a prognostic molecular biomarker of lung cancer and had the abilities to promote malignancy in lung cancer [9]. LncRNA FEZF1-AS1 plays crucial roles in numerous cancers, such as gastric cancer, colorectal carcinoma, lung cancer, nasopharyngeal carcinoma and glioblastoma [10–14]. Wang et al. [15] demonstrated that FEZF1-AS1 silencing inhibited HCC cell epithelial-mesenchymal transition (EMT) via JAK2/STAT3 pathway. However, the mechanism remains unknown.

Evidence has identified that miRNAs are frequently deregulated in cancers and involve in cancer development by altering the expression of target genes [16, 17]. For instance, miR-143 was found to be downregulated in bladder cancer [18] and breast cancer [19]. LncRNAs have been shown to usually act as sponges of miRNAs and then contribute to the development of cancers [20]. Using the bioinformatics methods, miR-107 is shown to be a predict target of lncRNA FEZF1-AS1, but their interaction in HCC waits to be verified.

We aimed to detect the regulatory pattern of FEZF1-AS1 in HCC in this study.

## RESULTS

The HCC tumorigenesis always accompanied with alteration of genes, and growing evidence suggested that lncRNAs are critical for cancer procession [21]. To explore the expression profiles of lncRNAs in HCC, the Arraystar Human lncRNA Microarray was performed in 3 paired HCC tissues and the neighboring normal tissues. A prominent alteration in FEZF1-AS1 level was found in the lncRNA profile (Figure 1A, 1B). The expression level of FEZF1-AS1 was found to be upregulated in HCC tissues as compared to the adjacent normal liver tissues by qRT-PCR (Figure 1C). We then detected the FEZF1-AS1 expression level in HCC cell lines. FEZF1-AS1 showed a higher expression pattern in SUN-182 cells and a lower expression pattern in Hep3b cells among the 4 cells, SNU-182, SNU-398, SNU-449 and Hep3b (Figure 1D).

**Figure 1:** **FEZF1-AS1 level was elevated in HCC.** (**A**) Heat map showing the differently expressed lncRNAs in the tumor tissues and adjacent normal tissues from HCC patients. Genes shown in red were upregulated and genes shown in green were downregulated lncRNAs. (**B**) Volcano plot of the differently expressed lncRNAs in the tumor tissues and adjacent normal tissues from HCC patients. Genes on the right were upregulated and genes on the downregulated lncRNAs. (**C**) The relative expression level of FEZF1-AS1 in tumor tissues and the adjacent normal tissues was detected by qRT-PCR, ^*^P < 0.05. (**D**) The relative expression levels of FEZF1-AS1 in HCC cell lines were tested by qRT PCR, ^*^P < 0.05.

To investigate the role of FEZF1-AS1 in HCC, it was overexpressed and downregulated in SNU-398 and SNU-449 because these two cells showed moderate level of EFZF-AS1 among the 4 cells (Figure 1D). qRT-PCR was used to detect the FEZF1-AS1 expression (Figure 2A) and CCK8 assay was used to assess the cell proliferation. Overexpression or downregulation of FEZF1-AS1 promoted or suppressed cell proliferation of SNU-398 and SNU-449 cells (Figure 2B, 2C). The flow cytometry demonstrated that FEZF1-AS1 overexpression suppressed the apoptosis of SNU-398 and SNU-449 cells (Figure 2D–2F). The results of transwell chamber and wound healing assays showed that FEZF1-AS1 overexpression significantly enhanced the invasion (Figure 2G–2I) and migration (Figure 3A, 3B) of HCC cells, and downregulation of FEZF1-AS1 caused opposite results. It is believed that EMT is a main cause of cancer cell migration and invasion. Therefore, we assessed FEZF1-AS1 role in HCC cell EMT. Results of western blot showed that FEZF1-AS1 overexpression induced EMT in HCC cells with increased expression levels of ICAM1 and Vimentin and decreased expression level of E-cadherin (Figure 3C, 3D), while downregulation of FEZF1-AS1 decreased ICAM1 and Vimentin expression and increased E-cadherin expression.

**Figure 2:** **FEZF1-AS1 promoted the proliferation and invasion and inhibits the apoptosis of HCC cells.** (**A**) qRT-PCR was used to detect the expression of FEZF1-AS1 after cell transfection with sh-NC, sh-FEZF1-AS1, OE-NC and OE-FEZF1-AS1 or without, ^*^P < 0.05, ^#^*P* < 0.05. (**B**, **C**) CCK8 assay was used to determine the proliferation of SNU-398 and SNU-449 cells, ^*^P < 0.05, ^#^*P* < 0.05. (**D**–**F**) Flow cytometry was used to test the apoptosis of SNU-398 and SNU-449 cells, ^*^P < 0.05, ^#^*P* < 0.05. (**G**–**I**) Transwell chambers were used to assess the invasion of SNU-398 and SNU-449 cells, ^*^P < 0.05, ^#^*P* < 0.05.

**Figure 3:** **FEZF1-AS1 promoted the migration and EMT of HCC cells.** (**A**, **B**) Wound healing assay was adopt to detect the migration of SNU-398 and SNU-449 cells, ^*^P < 0.05, ^#^*P* < 0.05. (**C**, **D**) Western blot was used to detect the expression levels of EMT markers, E-cadherin, ICAM1 and Vimentin, ^*^P < 0.05, ^#^*P* < 0.05.

Previous clues demonstrated that lncRNA was a molecular sponge of miRNA to impair their roles in repression the expression of target genes [22]. Herein, we found that miR-107 was targeted by FEZF1-AS1 and the binding sites were calculated by bioinformatics toll RagRNA2.0 (Figure 4A). The interaction between FEZF1-AS1 and miR-107 was then verified by the luciferase reporter assay. Co-transfection with psiCHEK2-FEZF1-AS1-WT and miR-107 mimics dominantly repressed the luciferase activity as compared to the mimic-NC group in SNU-398 and SNU-449 cells (Figure 4B, 4C). No obvious difference in the luciferase activity was observed between psiCHEK2-FEZF1-AS1-MUT with miR-107 mimics and psiCHEK2-FEZF1-AS1-MUT with miR-NC mimics groups (Figure 4B, 4C). To identify the relationship between FEZF1-AS1 and miR-107, we assessed miR-107 expression in SNU-398 and SNU-449 cells. FEZF1-AS1 overexpression significantly reduced miR-107 expression level (Figure 4D). On the contrary, FEZF1-AS1 downregulation decreased miR-107 expression level (Figure 4E).

**Figure 4:** **FEZF1-AS1 negatively regulated the expression of miR-107.** (**A**) The putative binding sites of miR-107 in FEZF1-AS1. (**B**, **C**) The relative luciferase activity was evaluated by luciferase gene reporter assay following cell transfection with pmirGlo-FEZF1-AS1-WT (wild type) or pmirGLo-FEZF1-AS1-MUT (mutant type) and miR-107 mimic or mimic-NC into SNU-398 and SNU-449 cells, ^*^P < 0.05. (**D**) The expression of miR-107 was assessed after downregulation of FEZF1-AS1 in SNU-398 and SNU-449 cells by qRT PCR, ^*^P < 0.05. (**E**) The expression of miR-107 was tested after overexpression of FEZF1-AS1 by q-RT-PCR, ^*^P < 0.05.

A previous study demonstrated that miR-107 involved in osteosarcoma by targeting Wnt/β-catenin pathway [23]. To explore whether FEZF1-AS1 targeted the miR-107/Wnt/β-catenin axis, we also assessed miR-107 and β-catenin levels in HCC. Compared to the adjacent normal liver tissues, miR-107 expression level was decreased and β-catenin expression level was increased in HCC tissues (Figure 5A, 5B). Then, miR-107 was overexpressed in SNU-398 and SNU-449 cells to assess its effect on the Wnt/β-catenin pathway. Western blot showed that miR-107 overexpression obviously suppressed the β-catenin and wnt3a expressions but enhanced the p-Gsk3β expression in SNU-398 and SNU-449 cells (Figure 5C–5F). To identify the involvement of Wnt/β-catenin signaling, the rescue assay was carried out. CCK8 assay showed that β-catenin overexpression significantly rescued the proliferation inhibition caused by FEZF1-AS1 shRNA in SNU-398 and SNU-449 cells (Figure 5G, 5H). The flow cytometry result showed that downregulation of FEZF1-AS1 enhanced cell apoptosis, while overexpression of β-catenin inhibited cell apoptosis in SNU-398 and SNU-449 cells (Figure 5I–5K). Also, upregulation of β-catenin promoted cell invasion (Figure 5L–5N) and migration (Figure 6A, 6B) which were inhibited by sh-FEZF1-AS1. Furthermore, western blot displayed that β-catenin overexpression increased ICAM1 and Vimentin expression levels which were suppressed by sh-FEZF1-AS1, and decreased E-cadherin expression level which was enhanced by sh-FEZF1-AS1 (Figure 6C, 6D).

**Figure 5:** **Downregulation of FEZF1-AS1 inhibited the proliferation and invasion of HCC cells by targeting miR-107/Wnt/β-catenin axis.** (**A**, **B**) The expression levels of miR-107 and β-catenin mRNA in HCC tissues and adjacent normal tissues were determined using qRT-PCR. (**C**–**F**) The relative expression levels of β-catenin, wnt3a and/or p-GSK3β were detected by qRT-PCR and western blot after cell transfection with mimic-NC and mimic-miR-107, ^*^P < 0.05. SNU-398 and SNU-449 cells were divided into three groups, sh-NC + OE-NC, sh–FEZF1-AS1 + OE-NC, and sh–FEZF1-AS1 + OE-β-catenin and submitted to the following assays. (**G**, **H**) Cell proliferation was detected by CCK8 assay, ^*^P <0 .01, sh–FEZF1-AS1 + OE-NC group vs. sh-NC + OE-NC group; ^#^*P* < 0.05, sh-FEZF1-AS1 + OE-β-catenin group vs. sh–FEZF1-AS1 + OE-NC group. (**I**–**K**) Cell apoptosis was detected by flow cytometry, ^*^P < 0.01, sh–FEZF1-AS1 + OE-NC group vs. sh-NC + OE-NC group; ^#^*P* < 0.05, sh-FEZF1-AS1 + OE-β-catenin group vs. sh–FEZF1-AS1 + OE-NC group. (**L**–**N**) Cell invasion was accessed by transwell chamber assay, ^*^P < 0.01, sh–FEZF1-AS1 + OE-NC group vs. sh-NC + OE-NC group; ^#^*P* < 0.05, sh-FEZF1-AS1 + OE-β-catenin group vs. sh–FEZF1-AS1 + OE-NC group.

**Figure 6:** **Downregulation of FEZF1-AS1 inhibited the migration and EMT of HCC cells by targeting miR-107/Wnt/β-catenin axis.** SNU-398 and SNU-449 cells were divided into three groups, sh-NC + OE-NC, sh–FEZF1-AS1 + OE-NC, and sh–FEZF1-AS1 + OE-β-catenin and submitted to the following assays. (**A**–**B**) Cell migration was detected by using the wound healing assay, ^*^P < 0.01, sh–FEZF1-AS1 + OE-NC group vs. sh-NC + OE-NC group; ^#^*P* < 0.05, sh-FEZF1-AS1 + OE-β-catenin group vs. sh–FEZF1-AS1 + OE-NC group. (**C**–**D**) The expression of EMT markers (E-cadherin, ICAM1 and Vimentin) were measured by western blot, sh-FEZF1-AS1 group vs sh-NC group, ^*^P < 0.01, sh–FEZF1-AS1 + OE-NC group vs. sh-NC + OE-NC group; ^#^*P* < 0.05, sh-FEZF1-AS1 + OE-β-catenin group vs. sh–FEZF1-AS1 + OE-NC group.

To verify the function of FEZF1-AS1 in HCC *in vivo*, SUN-398 cells with FEZF1-AS1 stable downregulation and/or β-catenin stable overexpression were transplanted into nude mice. Figure 7A showed the histopathological changes of the mice tissues and no cachexia was found after the nude mice were sacrificed. Downregulation of FEZF1-AS1 inhibited tumor growth with smaller volumes and less weights as compared with the sh-NC or normal saline group, whereas overexpression of β-catenin rescued the reduction of the tumor growth caused by shFEZF1-AS1 (Figure 7B, 7C). Additionally, FEZF1-AS1, wnt3a, β-catenin, ICAM1 and Vimentin expressions were repressed and E-cadherin and miR-107 levels were increased in the sh-FEZF1-AS1 group, whereas these tendencies were neutralized by β-catenin overexpression (Figure 7D, 7E).

**Figure 7:** **Downregulation of FEZF1-AS1 inhibited the tumor growth *in vivo* by targeting miR-107/Wnt/β-catenin axis.** SNU-398 cells were divided into four groups, normal saline group, sh-NC group, sh–FEZF1-AS1 group, and sh–FEZF1-AS1 + OE-β-catenin group. (**A**) HE staining was used to analyze of histopathological changes of mice tumor tissues. (**B**, **C**) The tumor volume and weight were detected after the mice were euthanized. (**D**) qRT-PCR was used to detect the expression of FEZF1-AS1 and miR-107 in mice tumor tissues. (**E**) Western blot was used to test the expression levels of wnt3a, β-catenin, E-cadherin, ICAM1 and Vimentin in mice tumor tissues. ^*^P < 0.01, sh–FEZF1-AS1 group vs. sh-NC group; ^#^*P* < 0.05, sh-FEZF1-AS1 + OE-β-catenin group vs. sh–FEZF1-AS1 group.

## DISCUSSION

HCC is a malignant cancer which is characterized by low survival rate [24]. Although great progress has been made in improving the therapeutic method of HCC in the past years, the efficacy is still unsatisfied. It’s important to investigate the oncogenic mechanisms in HCC. We proved in this study that FEZF1-AS1 had a high expression level in HCC. Also, we found that FEZF1-AS1 contributed to the malignant alterations of HCC via targeting miR-107/Wnt/β-catenin axis, as well as EMT, which is a main cause of cancer metastasis [25].

It was believed that lncRNAs played vital roles in HCC metastasis [26]. EZF1-AS1 is dysregulated in several cancers and contributes to carcinogenesis by targeting miRNAs or specific signaling pathway [13, 27–29]. Previous studies demonstrated that FEZF1-AS1 had an impact on the proliferation and invasion of HCC cells [15, 30]. Herein, we confirmed a high expression pattern of FEZF1-AS1 in HCC and FEZF1-AS1 overexpression promoted proliferation, migration and invasion of HCC cells. Further, we found miR-107 was another target of FEZF1-AS1 in HCC. From the luciferase gene reporter and qRT-PCR assays, we observed that FEZF1-AS1 could bind to and negatively regulate the expression of miR-107 in HCC.

MiRNAs play vital roles in controlling cell proliferation, apoptosis, migration and invasion. Dysfunction of miRNAs contributes to the occurrence and development of cancers [31]. MiR-107, a widely studied miRNA, was believed to be implicated in the development of many kinds of cancers. However, miR-107 function is controversial. For instance, some researched identified that miR-107 was a tumor suppressor in gastric cancer, NSCLC, breast cancer and bladder cancer [32–35], but some found that miR-107 was an oncogene in gastric cancer, bladder cancers and breast cancer by targeting different pathway [36–38]. Wang et al. [39] found that miR-107 could inhibit cell proliferation in HCC by binding to the 3'-untranslated region of HMGA2. In contrast, some studies demonstrated that miR-107 promoted HCC cell proliferation [40]. We found that miR-107 level was downregulated in HCC. miR-107 upregulation leaded to a significant inhibition in Wnt/β-catenin signaling with decreased expressions of β-catenin and wnt3a and an increased level of p-GSK-3β. However, miR-107 was identified to inhibit cell proliferation, colony-forming ability and tumorigenicity in osteosarcoma, with increased expression level of β-catenin [23]. We speculate that different cell contents maybe a main cause of the different roles of miR-107 plays in regulating β-catenin expression.

Furthermore, we explored whether Wnt/β-catenin signaling was regulated by FEZF1-AS1 in HCC. We found that β-catenin overexpression greatly enhanced cell proliferation and metastasis in HCC which were inhibited by FEZF1- AS1 downregulation. This result suggested that downregulation of FEZF1-AS1 inhibited HCC progression through inhibiting the Wnt/β-catenin pathway. However, miR-107 role in this process is not clear and we intend to clarify it in our further study.

As a whole, our study identified that FEZF1-AS1 accelerated the malignant behavior of HCC via miR-107/Wnt/β-catenin axis.

## MATERIALS AND METHODS

### Tissue obtainment

HCC tissues and the adjacent normal liver tissues were harvested from HCC patients in Shanghai Jiao Tong University Affiliated Sixth People’s Hospital between 2013 and 2015. Patients participated in this study received no other therapeutic method before surgery. This study was conducted in accordance with the World Medical Association Declaration of Helsinki and was approved by the Research Ethics Committee of Shanghai Jiao Tong University. Informed consent was written by each patient.

### Cell culture and transfection/infection

Hep3b, SNU-182, SNU-398 and SNU-449 cell lines were obtained from the American Type Culture Collection (ATCC, VA, USA). Cells were cultured in DMEM solution (Thermo Fisher scientific, NYC, USA), with 10% fetal bovine serum (FBS, Gibco, CA, USA) and 1% penicillin/streptomycin (Invitrogen, CA, USA).The shRNA used to knockdown FEZF1-AS1 (sh-FEZF1-AS1), the mimic used to upregulate miR-107 (mimic-miR-107), the plasmid used to overexpress FEZF1-AS1 (OE-FEZF1-AS1) and the lentivirus vector used to overexpress β-catenin (OE-β-catenin), as well as the negative controls (NC) were produced by GenePharma Co., LTD (Shanghai, China). Cells were transfected with mimic-NC, mimic-miR-107, OE-FEZF1-AS1 or OE-NC by using of Lipofectamine 2000 (Invitrogen, Carlsbad, CA, USA) according to the instruction. Other lentivirus vectors were infected into cells using polybrene and then incubated with puromycin and/or G418 for two weeks.

### Cell growth and apoptosis assay

The cell proliferation was tested by CCK8 kit (Beyotime, Beijing, China). 96-well plates were used to seed the cells at a density of 2000 cell/cm^2^ and the cells were transfected/infected with plasmids/lentivirus after 24 hours of incubation at 37°C. Following 24, 48, 72, 96 or 120 hours of incubation after inoculation, 10 μl CCK8 solution was then added into each well. The cells were incubated for 2 hours. Then, the absorbance was measured by the reader (model 680; Bio-Rad, Hertfordshire, UK) at 450 nm. Flow cytometry was used to determine the apoptosis rates of cells which were transfected/infected with sh-FEZF1-AS1, OE-FEZF1-AS1, sh-NC, OE-NC, mimic-NC, and mimic-miR-107. Annexin V(FITC)/PI Apoptosis Detection Kit (BioLengen, CA, USA) was used according to the instruction.

### Wound healing assay and transwell assay

Cells were seeded into six-well plates in a density of 3000 cells/cm^2^. After cell transfection/infection with plasmids/lentivirus, wounds were scraped by tips. The distance of the wound was captured after 0 hour and 24 hours of incubation at 37°C by DM2500 bright field microscope (LEICA, Wetzlar, Germany). The migration distance was measured by Image J. Upper chamber was coated with matrigel. Cells were seeded in the density of 3000 cells/cm^2^. Bottom chamber was filled with DMEM with 10% FBS and 1% penicillin/streptomycin. 4% paraformaldehyde (PFA) was used to fix the invaded cells and crystal violet was used to stain the cells. The amount of invaded cells was counted by image J.

### Luciferase reporter assay

The wild and mutant forms of the luciferase reporters (psiCHEK2-FEZF1-AS1-WT, psiCHEK2-FEZF1-AS1-MUT) were synthesized to detect the correlation of FEZF1-AS1 and miR-107. SNU-398 and SNU-449 cells were seeded into 96-well plates followed by co-transfection of mimic-NC, mimic-miR-107, psiCHEK2-FEZF1-AS1-WT, psiCHEK2-FEZF1-AS1-MUT using Lipofectamine 2000 (Invitrogen). 48 hours later, Dual Luciferase Assay System (Promega, USA) was used to detect the relative luciferase activity.

### Western blot assay

Total protein was isolated using lysis buffer (Cell Signaling Technology) containing protease inhibitors (Pierce Biotechnology, Waltham, USA). Equal amounts of protein were loaded on a 10% SDS-PAGE gel. The polyvinylidene fluoride membranes were blotted with the following primary antibodies, including mouse anti-E-cadherin (Abcam, ab76055), mouse anti-ICAM1 (Abcam, ab2213), mouse anti-vimentin (Abcam, ab8978), rabbit anti-p-GSK3 β (Abcam, ab75745), rabbit anti-β-catenin (Abcam, ab16051), rabbit anti-wnt3a (Abcam, ab234099) and Mouse anti-GAPDH (Multi sciences, ab011-040).

After 1 h incubating with secondary antibodies, anti-Mouse IgG-HRP (Thermos, RA230188) and anti-Rabbit IgG-HRP (ab205718), the blots were visualized by the Alphalmager™ 2000 Imaging System (Alpha Innotech, San Leandro, USA). The band density was quantified using ImageJ.

### Real time PCR (qRT-PCR) assay

Total RNA was extracted by TRIzol extraction kit (Invitrogen, Carlsbad CA, USA). cDNA was synthesized using the ReverTra Ace qPCR RT kit (Toyobo, Osaka, Japan). qRT-PCR was performed on a 7300 RT-PCR System (Applied Biosystem, Foster City, USA). The sequences of the primers were as follows: FEZF1-AS1-forward: 5′-GCTTGGCATTAGGAGAGCCT-3′, FEZF1-AS1-reverse: 5′-GGCTTTTAATTTTCGGGGCGT-3′; miR-107-forward: 5′-TCAGCTTCTTTACAGTGTTGCC-3′, miR-107-reverse: 5′-TCTGTGCTTTGATAGCCCTGT-3′; wnt3a-forward: 5′-GTGTTCCACTGGTGCTGCTA-3′, wnt3a-reverse: 5′-CCCTGCCTTCAGGTAGGAGT-3′; β-catenin-forward: 5′-GAAGGGGCTGACGCTATTGA-3′, β-catenin-reverse: 5′-GCTCCCAAGGAACGTCATCA-3′; GAPDH-forward: 5′-CCACCCCCAATGTCTCTGTT-3′, GAPDH-reverse: 5′-ATGGATGAACGGCAATCCCC-3′.

### *In vivo* assay

A mouse xenograft model was established using male BALB/c nude mice (Shanghai Slac Laboratory Animal Company (Shanghai, China) at an age of six weeks. Animals were housed in a controlled environment (50% humidity, 23 ± 2°C, 12-h light-dark cycle) with free access to water and food. 2 × 10^6^ SUN-398 cells were stably transfected with sh-FEZF1-AS1 and/or OE-β-catenin and resuspended in 100 μL normal saline. Then, the cells were then injected subcutaneously in flanks of mice. Cells in normal saline served as negative control. Four weeks later, all animals were euthanized and tumor xenografts were harvested. Weight of tumors were measured. All experiments regarding animal handling were approved by the Animal Care and Use Committee of Shanghai Jiao Tong University Affiliated Sixth People's Hospital and performed following the Guide for the Care and Use of Laboratory Animals.

### Statistical analysis

All experiments were performed in triplicate and repeated three times. Data were analyzed by the SPSS software (version 24.0) and shown as mean ± standard deviation. Student’s *t*-test and one-way analysis of variance (ANOVA) were used for statistical comparisons between two groups or among multiple groups, respectively. A value of *p* < 0.05 was considered statistically significant.
